The article "Effect of Cyanotoxins on the Hypothalamic–Pituitary–Gonadal Axis in Male Adult Mouse" was retracted in 2024. Reasons: errors in the data; duplicated images; duplicated data; duplicate publication.

# Effect of Cyanotoxins on the Hypothalamic–Pituitary–Gonadal Axis in Male Adult Mouse

**DOI:** 10.1371/journal.pone.0106585

**Published:** 2014-11-06

**Authors:** Xiaolu Xiong, Anyuan Zhong, Huajun Xu

**Affiliations:** 1 Department of Endocrinology, the Affiliated Drum Tower Hospital, Nanjing Medical University, Nanjing, China; 2 Department of Respiratory Diseases, the Second Affiliated Hospital of Soochow University, Suzhou, China; 3 Department of Otolaryngology, Shanghai Jiao Tong University Affiliated Sixth People's Hospital, Otolaryngology Institute of Shanghai Jiao Tong University, Shanghai, China; Clermont Université, France

## Abstract

**Background:**

Microcystins LR (MC-LR) are hepatotoxic cyanotoxins that have been shown to induce reproductive toxicity, and Hypothalamic–Pituitary–Gonadal Axis (HPG) is responsible for the control of reproductive functions. However, few studies have been performed to evaluate the effects of MC-LR on HPG axis. This study aimed to investigate the MC-LR-induced toxicity in the reproductive system of mouse and focus on the HPG axis.

**Methods:**

Adult male C57BL/6 mice were exposed to various concentrations of MC-LR (0, 3.75, 7.50, 15.00 and 30.00 µg/kg body weight per day) for 1 to 14 days, and it was found that exposure to different concentrations of MC-LR significantly disturbed sperm production in the mice testes in a dose- and time-dependent manner. To elucidate the associated possible mechanisms, the serum levels of testosterone, follicle-stimulating hormone (FSH) and luteinizing hormone (LH) were assessed. Meanwhile, PCR assays were employed to detect alterations in a series of genes involved in HPG axis, such as FSH, LH, gonadotropin-releasing hormone (GnRH) and their complement receptors. Furthermore, the effect of MC-LR on the viability and testosterone production of Leydig cells were tested *in vitro*. Results: MC-LR significantly impaired the spermatogenesis of mice possibly through the direct or indirect inhibition of GnRH synthesis at the hypothalamic level, which resulted in reduction of serum levels of LH that lead to suppression of testosterone production in the testis of mice.

**Conclusions:**

MC-LR may be a GnRH toxin that would disrupt the reproductive system of mice.

## Introduction

Cyanobacterial blooms and the production of secondary metabolites cyanotoxins represent a serious public health hazard to humans and animals worldwide since the cyanotoxins can be accumulated in aquatic organisms and transferred to higher trophic levels [1], [2]. One of the most frequently studied cyanotoxins is the cyclic heptapeptide hepatotoxins called microcystins (MCs) due to their wide distribution and high toxicity. Up to now, more than 80 analogues of MCs have been identified, with microcystin-LR (MC-LR) being the most common and toxic [3]. Studies demonstrated that the mechanism of MCs toxicity is the potent inhibition of serine/threonine- specific protein phosphatases 1 and 2A (PP1 and PP2A), which then leads to the hyperphosphorylation of key control proteins that regulate tumor promotion or apoptosis [4]. MCs could also induce the production of reactive oxygen species (ROS) in cells which subsequently can trigger apoptosis or necrosis [5], [6]. It was reported that MCs accumulated mainly in liver and were known for their hepatotoxic effects [7]. Moreover, MCs could also accumulate in heart, kidney and embryo, resulting in toxicity to those organs [8].

Recently, several studies have demonstrated that MCs would exert negative effects on the male reproductive system and gonads are regarded as the second important target organs of MCs [9]. It was reported that MCs could accumulate in testis and induce rat testis cell apoptosis [10], MCs could also induce morphological damages, cause significant decrease of sperm quality [11], and decline of serum hormones such as testosterone, follicular stimulating hormone (FSH) and luteinizing hormone (LH) levels [12]. However, molecular mechanisms underlying such reproductive toxicity of MCs are still unclear.

A small subset of hypothalamic neurons expressing gonadotropin releasing hormone (GnRH), the gonadotrope cells in anterior pituitary and the gonads form an integrated system hypothalamus-pituitary-gonadal axis (HPG) that is responsible for the adequate secretion of male hormones and normal spermatogenesis [13]. The testes require stimulation by the pituitary gonadotropins such as luteinizing hormone (LH) [14] and follicle-stimulating hormone (FSH) [15], which are secreted in response to hypothalamic gonadotropin releasing hormone (GnRH) [16]. The effect of LH and FSH on germ cell development is mediated by the androgen and FSH receptors that are present on Leydig and Sertoli cells, respectively [17]. Whereas FSH acts directly on the germinal epithelium and stimulates Sertoli cells to support spermatogenesis, LH promotes the Leydig cells to secrete testosterone which boosts sperm production and virilization and provides feedback to the hypothalamus and pituitary to regulate GnRH secretion [18], [19].

To date, few studies have been performed to evaluate the effects of MCs on HPG axis. The aim of the present study was to investigate the MC-LR-induced toxicity in the reproductive system of mouse and focus on the HPG axis. The results demonstrated that exposure to different concentrations of MC-LR significantly disturbed sperm production in the mice testes. To elucidate the associated possible mechanisms, the serum levels of testosterone, FSH and LH were assessed. Meanwhile, PCR assays were employed to detect alterations in a series of genes involved in HPG axis, such as FSH, LH, GnRH and their complement receptors. Furthermore, the effect of MC-LR on the viability and testosterone production of Leydig cells were tested *in vitro*.

## Materials and Methods

### Animals

Adult male C57BL/6 mice (6 weeks old and weighed 18–22 g) were obtained from the Animal Center of Nanjing Medical University (Nanjing, China). Mice were individually housed in laminar flow cabinets under a specific pathogen-free environment with access to food and water ad libitum. The animals were acclimatized for 1 week before use, and maintained throughout at standard conditions: 50% relative humidity, 24°C±1°C) and 12∶12-h light-dark circle. This study was carried out in strict accordance with the recommendations of JiangSu Provincial Experimental Animal Manage Committee under Contract 2011–0069. All surgery was performed under sodium pentobarbital anesthesia, and all efforts were made to minimize suffering. All experimental procedures were conducted in conformity with institutional guidelines for the care and use of laboratory animals, and protocols were approved by the Institutional Animal Care and Use Committee in NANJING Medical College, jiangsu, China.

### MC-LR Exposure

Purified MC-LR (purity ≥ 98%) was purchased from Alexis Biochemicals (Lausen, Switzerland) and was dissolved in physiological saline solution (0.9% NaCl) for injection. The LD50 of MC-LR was determined by Dixon's up and down method for small samples as described previously [3]. Mice were randomized into five groups (n = 20 for each): *1*) 3.75 µg group, which received intraperitoneal injection (i.p.) of MC-LR at the dose of 3.75 µg/kg body weight per day (1/16 LD50); *2*) 7.50 µg group, which were intraperitonealy injected with 7.50 µg/kg body weight per day (1/8 LD50) of MC-LR; *3*) 15.00 µg group, which were intraperitonealy injected with 15.00 µg/kg body weight per day (1/4 LD50) of MC-LR; *4*) 30.00 µg group, which were intraperitonealy injected with 30.00 µg/kg body weight per day (1/2 LD50) of MC-LR; *5*) Control group, which received i.p. injection of the same volume of 0.9% saline solution. Mice in the five groups were sacrificed at 1, 4, 7, 14 days postinjection, respectively. Five mice were sacrificed at each time point. Mice were anesthetized with 1% sodium pentobarbital (100 mg/kg intraperitoneally), then blood was collected by cardiac puncture with a heparinized syringe, the hypothalamic, pituitary and testis tissues were rapidly removed, weighed, and perfused with ice-cold PBS (pH 7.4). Part of the tissues were stored in RNA later reagent (Qiagen, Tokyo) at 4°C for extraction of RNA, and the remaining samples were snap-frozen in liquid nitrogen and stored at −80°C until required. Serum was immediately collected by centrifugation (4,000 rpm at 4°C) and stored at −20°C.

### Hormone Measuring Assay

Blood was collected by cardiac puncture with a heparinized syringe and serum was immediately collected by centrifugation (4,000 rpm at 4°C) and stored at −20°C for further analysis. Serum levels of testosterone, folliclestimulating hormone (FSH) and luteinising hormone (LH) were determined using ELISA kits (Assay Designs, Ann Arbor, MI, and Amersham Biosciences) according to the manufacturer's instructions. All samples were tested in triplicate. The sensitivities of the mouse testosterone, FSH and LH assays were 0.002 ng/ml, 0.4 IU/L and 0.3 IU/L, respectively. The interassay coefficient of variation was less than 10% for all assays.

### Evaluation of Epididymal Sperm

After the mice were treated with MC-LR, at the indicated time point, the epididymides were removed and minced in 1.5 ml of KSOM and 3% BSA for 30 min at 37°C, to release sperm into the medium. Spermatozoa were extracted from the whole epididymis, and the total sperm count was assessed in the final suspension by using a hemacytometer.

### Real-time quantitative PCR analysis

Total RNA was isolated from tissues using Trizol reagent (Invitrogen, Carlsbad, CA, USA) and cDNA was synthesized from 2 µg of total RNA using Moloney murine leukemia virus reverse transcriptase (MMLV) (Promega, Madison, WI, USA). The PCR products were analyzed by electrophoresis on 1.5% agarose gel. The electrophoretic products were photographed using a gel imaging system. Real-time quantitative PCR using SYBR Premix (DRR041A, TaKaRa, Japan) was performed according to the producer's specifications. Amplifications were performed in a LightCycler machine (Roche Diagnostics, Basel, Switzerland) following the manufacturer's instructions. A uniform amplification of the products was rechecked by analyzing the melting curves of the amplified products. 18s rRNA was used as an endogenous control for each sample. All samples were assayed in triplicate. The primer sequences used to amplify specific target genes were listed in Table 1.

**Table 1:** Primer sequences used for real-time polymerase chain reaction analysis.

Gene	Primer sequence	Product size(bp)	Annealing Temperature (°C)	Cycles
FSHr	(f) 5′-TGCTACACCCACATCTACCT-3′	307	60	32
	(r) 5′-GCACCTCATAACAGCCAAAC-3′			
LHr	(f) 5′-ATTCAGACGCTCATCGC-3′	370	56.6	38
	(r) 5′-GCCAAATCAACACCCTAA-3′			
GnRHr	(f) 5′-ATCCCTTTGACTTTCACATCC-3′	184	61	35
	(r) 5′-CACCTCCTTGCCCATCTC-3′			
FSHβ	(f) 5′-TCCCTCCATCCATACTGT-3′	463	56	32
	(r) 5′-GCTTGGTTACTACCTCCTG-3′			
LHβ	(f) 5′-CGGCCTGTCAACGCAACT-3′	110	60	40
	(r) 5′-GGCAGTACTCGGACCATGCT-3′			
GnRH1	(f) 5′-ATCCCTTTGACTTTCACATCC-3′	184	61	32
	(r) 5′-CACCTCCTTGCCCATCTC-3′			
Kiss-1	(f) 5′-CCACCTACAACTGGAACTCCTTCG-3′	110	60	34
	(r) 5′-CCCTGCCTTGGCCTCTACAATC-3′			
Gpr54	(f) 5′-GGCTCCGTCCAACGCTTCAG-3′	174	64	32
	(r) 5′-TGTGCTTGTGGCGGCAGATA-3′			
18s rRNA	(f) 5′-AGGGGAGAGCGGGTAAGAGA-3′	241	60	27
	(r) 5′-CACCTCCTTGCCCATCTC-3′			

Abbreviation: FSH: folliclestimulating hormone, LH: luteinising hormone, GnRH: gonadotropin releasing hormone, RNA: ribonucleic acid.

### Isolation and culture of primary Leydig cells

After all mice were sacrificed by exsanguination under anaesthesia. The sterile testes were dissected and washed thrice in 4°C PBS. Epididymis, visible vessels, fat and other connective tissues were carefully removed from testes with microscissors. The tunica albuginea was then dissected out, and pair of testes from each mouse were incubated in a 50-ml centrifuge tube containing 5 ml of 0.03% collagenase NB4 (Serva, Heidelberg, Germany). The testes were digested for 15 min at 37°C with vibration at 150 rpm as the first step. The supernatant was discarded. Another 5 ml of fresh collagenase NB4 was added into the centrifuge tube, and the cell pellet was digested for another 15 min at 37°C as the second step, during which the vibration speed was lowered from 150 to 130 rpm. Cells in the supernatant were then centrifuged and resuspended in low glucose DMEM (Gibco, Carlsbad, CA, USA) with 10% fetal bovine serum (FBS; Gibco, Grand Island, NY, USA) for seeding. Cultures were performed in a humidified incubator at 37°C under a 5% CO_2_ atmosphere. Cells from the supernatant were examined by trypan blue dye exclusion for viability and then analyzed for Leydig cell purity with 3β-HSD histochemical staining.

### Cell viability assay

Cell viability was measured by using Cell Counting Kit-8 (Dojindo, Kumamoto, Japan) according to the manufacurer's instructions. Exponentially growing Leydig cells were digested by 0.25% trypsin for 1–2 min, and washed thrice with PBS. Then 2×10^5^ cells in 100 µl culture medium were plated in 96-well plates followed 12 hours later by addition of MC-LR at the final concentration of 0, 1.0, 10.0, 100.0, 250.0, 500.0, 750.0 and 1000.0 nmol/L. 48 h later, the medium was aspirated and each well was added with 100 µl serum-free DMEM and 10 µl CCK-8 and incubated at 37°C for 1.5 hours. Absorbance was measured at 450 nm with a reference wavelength of 630 nm on a spectrophotometer (Molecular Devices, Sunnyvale, CA). Cell viability was assessed as percent cell viability in terms of untreated control cells, which were determined for each concentration by use of the following equation: %viability  =  OD_experiment/ODcontrol_ ×100%. Control cells were considered as 100% viable. All experiments were repeated in six times.

### Testosterone levels produced by Leydig cells *in vitro*

Leydig cells were cultured with MC-LR at the final concentration of 0, 1.0, 10.0, 100.0, 250.0, 500.0, 750.0 and 1000.0 nmol/L for 48 hours, then the supernatants were collected to analyze the testosterone levels by using an ELISA kit (Assay Designs, Ann Arbor, MI, and Amersham Biosciences) according to the manufacturer's instructions. All samples were tested in triplicate.

### Statistical analysis

GraphPad Prism version 5.03 (GraphPad, San Diego, CA, USA) was used for all statistical analyses. All data are expressed as mean ± SEM. Differences between groups were analyzed by a 2-tailed Student's paired t-test for single comparisons and by one-way ANOVA with LSD *post-hoc* test for multiple comparisons. Bonferroni's correction was used to adjust for multiple comparisons. A *P* value <0.05 was considered to be statistically significant.

## Results

### Effect of MC-LR on the Sperm production

To determine whether MC-LR administration affects the spermatogenesis of mice, mice were treated with MC-LR at various concentrations (0, 3.75, 7.50, 15.00 and 30.00 µg/kg body weight per day), at the indicated time point, the epididymides were removed and minced to release sperm into the medium. the sperm quantity was measured using a hemacytometer. As shown in Fig. 1, increasing MC-LR concentration and treatment time resulted in a progressive inhibition of spermatogenesis. At day 1, there was no difference of the epididymal sperm production between various concentrations of MC-LR and the control group ((0 µg/kg/day MC-LR). However, treatment with MC-LR for more than 4 days resulted in a significant dose- and time-dependent reduction in epididymal sperm production. The first significant reduction was observed at the concentration of 15.00 µg/kg/day MC-LR after administration for 4 days, with an inhibition of 20.48% (*P*<0.05). The low concentration of MC-LR (3.75 µg/kg/day) showed no effect on the sperm production even extended the treatment time. These results demonstrated that MC-LR had a potent inhibitory effect on the spermatogenesis of mice.

**Figure 1:** Effect of MC-LR on sperm production. After the mice were treated with MC-LR at various concentrations (0, 3.75, 7.50, 15.00 and 30.00 µg/kg body weight per day), at the indicated time point, the epididymides were removed and minced to release sperm into the medium. Spermatozoa were extracted from the whole epididymis, and the total sperm count was assessed in the final suspension using a hemacytometer. Results represent the means ± SEM of five mice. *, P<0.05; #, P<0.01; §, P<0.005 versus control group (MC-LR 0 µg/kg body weight per day).

### Effect of MC-LR on the hormone levels

Testosterone is important for spermatogenesis and LH signaling is critical for testosterone production from the Leydig cells. To analyze whether significantly reduced spermatogenesis was associated with the testosterone levels, the serum testosterone was assessed. As shown in Fig. 2A, serum testosterone was significantly suppressed in a dose- and time-dependent manner after treatment of MC-LR for 4 days. The low concentration of MC-LR (3.75 µg/kg/day) did not affect the serum testosterone level during the experiment time. It was initially observed that after administration of 15.00 µg/kg/day MC-LR for 4 days, the testosterone was decreased by 31.25% (Fig. 2A, P<0.05). These data were consistent with the previous results that treatment of mice with MC-LR for more than 4 days significantly inhibited the spermatogenesis of mice. Similarly, the serum LH levels (Fig. 2B) varied in a dose- and time-dependent manner in response to MC-LR treatment as well. However, the serum FSH levels were not changed by the MC-LR administration (Fig. 2C). Taken together, these results indicated that inhibited serum testosterone and LH induced by MC-LR contributed to the impaired spermatogenesis of mice treated with MC-LR.

**Figure 2:** Effect of MC-LR on hormone levels. Mice were treated with various concentrations of MC-LR (0, 3.75, 7.50, 15.00 and 30.00 µg/kg body weight per day), at the indicated time point, serum testosterone (A), folliclestimulating hormone (FSH) (B) and luteinising hormone (LH) (C) were measured by ELISA, *respectively*. Data represent the means ± SEM from five mice. *, P<0.05; #, P<0.01; §, P<0.005 versus control group (MC-LR 0 µg/kg body weight per day).

### Effect of MC-LR on the viability and Testosterone levels of Leydig cells *in vitro*

The primary Leydig cells were isolated from the mice testis, the cell viability was around 90% by trypan blue detecting. The isolated cells showed a uniform epithelial-like shape. After 7 days of culture, 90% of the cells were positive for 3β-HSD histochemical staining, which indicated the purity of the isolated Leydig cells. To test the effect of MC-LR on Leydig cell viability, Leydig cells were cultured with MC-LR at the final concentration of 0, 1.0, 10.0, 100.0, 250.0, 500.0, 750.0 and 1000.0 nM. The cell viability was assessed by the WST-8 assay 24 h later. As shown in **Fig. 3A**, no significant difference in cell viability was observed between various concentrations of MC-LR and the control group (0 nM MC-LR). Moreover, the Leydig cell-derived testosterone levels were measured after MC-LR treatment. However, MC-LR showed no effect on the testosterone levels *in vitro* (Fig. 3B).

**Figure 3:** Effect of MC-LR on Leydig cell viability after 48 h incubation. 2×10^5^ Leydig cells in 100 µl culture medium were plated in 96-well plates followed 12 hours later by addition of MC-LR at the final concentration of 0, 1.0, 10.0, 100.0, 250.0, 500.0, 750.0 and 1000.0 nmol/L. 48 h later, the effect of MC-LR on cell viability was determined by the CCK-8 assay as described in Materials and Methods. Results represent the means ± SEM of six samples. Effect of MC-LR Testosterone levels produced by Leydig cells *in vitro*. Leydig cells were cultured with MC-LR at the final concentration of 0, 1.0, 10.0, 100.0, 250.0, 500.0, 750.0 and 1000.0 nmol/L for 48 hours, then the supernatants were collected to analyze the testosterone levels by using an ELISA kit. Results represent the means ± SEM of three samples.

### Effect of MC-LR on the gene expression of FSHR and LHR in the testis of mice

To investigate the possible effects of MC-LR on the expression of two gonadotropin receptors FSHR and LHR in the testis, mice were intraperitonealy injected with MC-LR at the concentrations of 0, 3.75, 7.50, 15.00 or 30.00 µg/kg body weight per day, at the indicated time point, the LHr and FSHr mRNA were detected with RT-PCR. 18s rRNA was used as an internal control for equal loading of samples. As shown in Fig. 4, no significant difference in the expression of *FSHR* or *LHR* was observed between the MC-LR -treated and vehicle mice by semiquantitative RT-PCR analysis.

**Figure 4:** Effect of MC-LR on gene expression of LHr and FSHr. Mice were treated with various concentrations of MC-LR (0, 3.75, 7.50, 15.00 and 30.00 µg/kg body weight per day), at the indicated time point, the LHr and FSHr mRNA were detected with RT-PCR. 18s rRNA was used as an internal control for equal loading of samples. Representative blots shown were from 6 mice.

### Effect of MC-LR on GnRHR, FSHβ and LHβ mRNA levels in the pituitary of mice

To determine whether MC-LR affects the hypothalamo-pituitary-gonadal (HPG) axis, the mRNA the expression of the gonadotropin genes *LHβ*, *FSHβ* and *GnRHR* in the pituitary were analyzed by RT-PCR after mice were intraperitonealy given with various concentrations of MC-LR. As shown in Fig. 5A, there were no significant differences of *GnRHR* and *FSHβ* between the MC-LR -treated and control by semiquantitative RT-PCR analysis. However, treatment of MC-LR for more than 4 days resulted in a significant dose- and time-dependent reduction in the expression of *LHβ* mRNA level. The results were further confirmed by quantitative real-time RT-PCR (Fig. 5B). These findings were consistent with the changes of serum hormone levels after MC-LR treatment.

**Figure 5:** Effect of MC-LR on gene expression of GnRHr, FSHβ and LHβ. Mice were treated with various concentrations of MC-LR (0, 3.75, 7.50, 15.00 and 30.00 µg/kg body weight per day), at the indicated time point, the GnRHr, FSHβ and LHβ mRNA were detected by RT-PCR or quantitative real-time RT-PCR. 18s rRNA was used as an internal control for equal loading of samples. Results represent means ± SEM of 6 mice. *, P<0.05; #, P<0.01; §, P<0.005 versus control group (MC-LR 0 µg/kg body weight per day).

### Effect of MC-LR on GnRH1, Kiss-1 and Gpr54 mRNA levels in the hypothalamus of mice

To further investigate whether MC-LR affects the HPG axis, the mRNA the expression of *GnRH1, Kiss-1* and *Gpr54* in the hypothalamus were analyzed by RT-PCR after mice were treated with MC-LR. Kiss1 mRNA levels in the hypothalamus did not vary significantly among the different treatment groups (Fig. 6A). No significant changes were observed in the kisspeptin receptor Gpr54 mRNA expression profile in hypothalamus of the mice at any time after MC-LR treatment (Fig. 6A). However, with regard to the changes in *GnRH1* mRNA levels, there was a similar trend of GnRH1 variation (Fig. 6A) to that of LHβ mRNA level (Fig. 5A). Comparing in this way, the two figures for the two mentioned variables, quantitative real-time RT-PCR assay further confirmed that administration of MC-LR significantly decreased the *GnRH1* mRNA levels in a dose- and time-dependent manner as compared with the group received the vehicle control saline treatment (Fig. 6B).

**Figure 6:** Effect of MC-LR on gene expression of GnRh1, Kiss-1 and Gpr54. Mice were treated with various concentrations of MC-LR (0, 3.75, 7.50, 15.00 and 30.00 µg/kg body weight per day), at the indicated time point, the Gnrh1, Kiss-1 and Gpr54 mRNA were detected with RT-PCR. RT-PCR or quantitative real-time RT-PCR. 18s rRNA was used as an internal control. Data represent means ± SEM of 6 mice. *, P<0.05; #, P<0.01; §, P<0.005 versus control group (MC-LR 0 µg/kg body weight per day).

## Discussion

The exposure to MCs has been reported to induce reproductive toxicity to animals [11], however, the underlying mechanisms of reproductive toxicity of MCs are still unclear. In the present study, we demonstrated that exposure to different concentrations of MC-LR significantly disturbed sperm production in the mice testis, which was associated with the suppression of GnRH expression that impaired the testosterone synthesis ability.

Spermatogenesis is a complex process by which the spermatogonia mature gradually to spermatozoa through a series of events involving mitoses, meiosis and cellular differentiation [21]. The spermatogenesis process was considered critically dependent on the high intratesticular testosterone levels induced by the two pituitary gonadotropins, LH and FSH [22]. LH and FSH are heterodimers consisting of a common *α*-subunit noncovalently linked to a hormone-specific *β*-subunit. The latter confers biologic specificity to the two ligands and determines the levels of functional FSH and LH [23]. LH stimulates testosterone production by Leydig cells whereas FSH stimulates the Sertoli cells to regulate spermatogenesis by secreting various factors that will affect Leydig cell function [20]. The exposure to many environmental toxicants leads directly to a remarkable decline in spermatogenesis function and fertility of animals and humans [12]. Several recent studies have demonstrated the reproductive toxicity of MCs to mammals [9], [11], [24]. It has been reported that exposure to MC-LR affects male reproductive organs and reduction of sperm number in mice [12], [24]. In the present study, our results indicated that spermatogenesis was significantly inhibited in mice treated with MC-LR compared with the vehicle-treated mice, and MC-LR exposure significantly decreased serum testosterone and LH level while FSH concentrations kept unchanged. As the secretion of testosterone is regulated by LH, the decreased serum testosterone level was as a result of low LH levels in mice. Although intratesticular testosterone levels were shown to be significantly higher than serum testosterone levels [25], the intratesticular testosterone highly correlated with serum testosterone [26]. Thus, the decreased serum testosterone level indicated the inhibited testosterone production in the testis which lead to impaired spermatogenesis. Recent studies showed that MCs accumulated in testis, and exerted toxic effects on reproductive system [10]. However, the *in vitro* experiments in the present study demonstrated that exposure to MC-LR had no effect on the viabilities and testosterone levels of Leydig cells which locates in the testicular interstitium and are the primary cells that synthesize and secrete testosterone in adult male animals. Thus, our data suggested that MC-LR did not affect testosterone synthesis by directly damaging Leydig cells.

The biological action of LH and FSH in gonadal tissue is mediated via membrane receptors for LH (LHR) and FSH (FSHR), respectively [27]. In the male animals, LHR is maily expressed in testicular. Leydig cells and on ligand binding, it stimulates androgen production. FSH binds to receptors FSHR on the surface of Sertoli cells and functions in concert with testosterone to promote the spermatogenesis function [18], [19]. In the present study, there was no effect of MC-LR i.p. injection on the plasma level of FSH in mice, which was later confirmed by the RT-PCR results which showed MC-LR did not affect the mRNA expression of *FSHβ* in the pituitary and *FSHR* in the testis, indicating that there was a normal interaction between *FSHR* and *FSH* in the testis of MC-LR-treated mouse, and MC-LR was not able to inhibit the FSH synthesis and secretion. However, the levels of *LHβ* transcripts in MC-LR-treated mice were suppressed with decreasing the LH synthesis in the pituitary, whereas the *LHR* expression was not affected, suggesting that Leydig cells in testis received the impaired LH pulse via LHR, which lead to inhibited production of testosterone.

The hypothalamic-pituitary-gonadal (HPG) axis is fundamental to the control of reproductive functions, whose main actor is the hypothalamic gonadotropin releasing hormone (GnRH) [13]. The decapeptide GnRH is produced by a subset of neurons with a scattered distribution throughout the basal forebrain and released into the hypophyseal portal vasculature from axon terminals at the median eminence [28]. Intermittent GnRH secretion from the hypothalamus acts upon the GnRH receptor (GnRHR) in the anterior pituitary to regulate the production and secretion of gonadotropins including LH and FSH that in turn regulate development and activity of the testes [29]. The pituitary requires pulsatile stimulation by GnRH to synthesize and release the gonadotropins LH and FSH, in turn, the feedback from gonadotropins finely modulate the GnRH release [30]. Moreover, the GnRH secretion depends on the activation of the GPR54 [31], located on the surface of the GnRH neurons and stimulated by the peptide kisspeptin which is a product of the *Kiss-1* gene [32]. In the present study, alterations in the GnRH1 gene expression were observed after i.p. injection of MC-LR, suggesting that MC-LR affected the reproductive system by means of actions at the level of the hypothalamus through modulation of GnRH synthesis and / or release. A lower GnRH secretion to the hypophyseal portal blood would result in the reduction of LHβ synthesis, which caused the decreasing testosterone production in the testis. GnRH could affect the GnRHR gene expression directly at the pituitary level. However, in the present study, the GnRHr mRNA levels kept unchanged. The mechanism awaits to be elucidated in our future study. In addition, no variations of GPR54 and Kiss-1 mRNA expression were observed in the study, indicating that MR-LR may not affect the GPR54/Kiss-1 regulation system directly.

The gonadotrope cell of the anterior pituitary plays a particularly critical role within the HPG axis system as the intermediary between the hypothalamic GnRH signal and the steroid hormone productivity of the gonads [33]. FSH and LH stimulate sex steroid production and secretion in the gonads. These molecules then feed back to the brain and pituitary to regulate the gonadotropins. In general, androgens (testosterone and dihydrotestosterone) have negative feedback effects primarily on the release of GnRH from the hypothalamus, which then suppresses both FSH and LH secretion [34]. When serum testosterone level is reduced, the GnRH synthesis and secretion increases followed by a subsequent rise in the synthesis and secretion of LH from the pituitary gland [34]. In the present study, MC-LR administration to mice resulted in a reduction in the serum testosterone concentration in a dose- and time- dependent manner. Intriguingly, the serum LH synthesis and secretion were reduced as well. Such phenomenon could be explained by the assumption that the possible increase in GnRH expression stimulated by the decreased testosterone level had been offset by the inhibited GnRH synthesis caused by exposure to MC-LR, which further demonstrate that the primary target of MC-LR is GnRH and MC-LR would disrupt the GnRH expression directly or indirectly.

Studies showed that MCs cannot readily diffuse through plasma membrane due to the high molecular weight and structure [2]. However, due to the cell specificity and organotropism of MC-LR, there should be some selective pathways of MC up-take. Recently, Fischer *et al*. [35] showed that MC-LR can be transported by different members of the organic anion transporting polypeptide superfamily (rodent: Oatps) and the OATP which is a multispecific transport system expressed in diverse cell types such as enterocytes, hepatocytes and renal epithelial cells [36] and organs including the heart, lung, brain and blood-brain-barrier [36]. We presumed that MC-LR would transport through the blood-brain-barrier into the hypothalamus to inhibit the GnRH expression, which resulted in downregulation of LHβ in the pituary that attenuates the testosterone synthesis in the testis, and finally the spermatogenesis was impaired. Thus, it was highly possible that GnRH was a direct or indirect target for MC-LR to damage the reproductive system of mice. However, the exact molecular mechanism for this is still unclear.

In conclusion, our results showed MC-LR significantly impaired the spermatogenesis of mice possibly through the direct or indirect inhibition of GnRH synthesis at the hypothalamic level, which resulted in reduction of serum levels of LH that lead to suppression of testosterone production in the testis of mice. Thus, MC-LR may be a GnRH toxin that would disrupt the reproductive system of mice.
